This article has been retracted.

# The Development and Realization of Digital Panorama Media Technology Based on VR Technology

**DOI:** 10.1155/2022/1023865

**Published:** 2022-04-28

**Authors:** Yake Qiu, Jingyu Tao

**Affiliations:** ^1^Department of Art and Design, Nanchang University, Nanchang, Jiangxi, 330031, China; ^2^Department of Humanities, Nanchang University, Nanchang, Jiangxi, 330031, China

## Abstract

The purpose of this paper is to understand the digital 3D multimedia panoramic visual communication technology based on virtual reality. Firstly, the key concepts and characteristics of virtual reality are introduced, including the development and application of digital three-dimensional panorama technology. Then, according to the theoretical research, some basic knowledge of 3D panoramic image Mosaic is introduced, including camera image modeling, image sharing, and image exchange. Finally, with the development of the virtual tour at the College of Normal University, the hardware of panoramic technology and the demand of panoramic image search have been expanded in the application. The design of panoramic Mosaic, panoramic image generation, and virtual tour school construction considers real-world issues. The innovation of this paper lies in that will be used by SketchUp8.0 software builds the geometry of 3d virtual scene and by the cylindrical panoramic images based on image of building 3 d virtual scene organic unifies in together and makes a panoramic image can be as the change of seasons in the real scene and real-time change, enhance the sense of the reality of the system and user immersive.

## 1. Introduction

Today, with the further development of cloud computing, Internet of Things, GIS, and other technologies, more and more applications choose to use these technologies to serve users, entering the era of software-as-a-service. Networked applications are the premise of the software-as-a-service era. Networked applications are widely used in the field of GIS, such as Baidu Maps, Google Maps, and Sky Maps. To realize the release and management of geographic information, especially now, The Street View service is in full swing and has become the focus of the development of various manufacturers. Its virtual three-dimensional scene and real on-site photos give users a sense of immersion, operation, and integration. But after all, such three-dimensionality is virtual and incalculable, Fake 3D. However, the real 3D display has shortcomings such as a large amount of data, cumbersome modeling process, and inconvenient data updating. How to make up for these shortcomings is the key to the current development [1]. The application of virtual reality technology in education is mainly reflected in the construction of a “digital campus.” The content mainly integrates campus culture, teaching staff, etc., showing the school's comprehensive strength in running a school. In form, it has developed from a traditional two-dimensional virtual campus to a three-dimensional virtual campus with a sense of reality, immersion, and greater interaction, which has played a positive role in the school's enrollment and publicity work and has also played a positive role in the school's digital construction [2] (Figure 1). Three-dimensional panoramic virtual reality technology (also called virtual reality) is a virtual reality technology of real scenes based on panoramic images. Panorama is to use a digital camera to shoot the real scene in a certain way when the viewpoint is fixed, rotate 360 degrees around the vertical axis according to a uniform angle, take one or more sets of photos according to the specific situation, stitch, adjust, and integrate the images in the computer, generate seamless panoramic images according to the expression classification, and realize the real scene restoration display mode of all-round interactive viewing through computer technology [1]. The three-dimensional panoramic display can give people a sense of proximity, a sense of being on the scene. When browsing online, the sense of presence directly affects the audience's effect of receiving information, thereby arousing the audience's interest and better information dissemination effect. The high-definition panoramic tour will give the audience a strong sense of presence.

This article through to Flex and PV3D integrated use of technology and builds the 3d virtual campus system based on panoramic images; the interaction of the system is good, in which the user can freely roam, and users can have a real immersive feeling, which had a profound influence on school's external publicity and has important application value.

## 2. Literature Review

Wang et al. used a pair of hyperboloid refractive mirrors and a camera lens to form a stereo panoramic vision system [3]. Tomoe et al. have also carried out pioneering research work in this area and proposed a design method that uses an ordinary camera to achieve an omnidirectional stereo vision. The design method is to process a pair of hyperboloid refracting mirrors into a single refracting mirror. The principle is similar to that of Koyasu's. Both devices have the advantage of compact structure [4]. Morra et al. designed a variety of point light source projection range meters, through the recognition of the point light source to achieve the depth information measurement of the object point [5]. This method can quickly obtain the three-dimensional information of the object point, but the amount of three-dimensional information obtained each time is small. Shen et al. designed a line structured light rangefinder, which allows the laser to generate a line light source through a cylindrical lens and rotates at a uniform speed through a stepping motor to sweep the beam across the surface of the object to be measured, thereby obtaining a series of images for information extraction and measurement [6]. Zhou et al. proposed to use a point laser to rotate at a high speed to form a conical laser plane and receive the panoramic light source information through the conical mirror and then analyzed the projection light source information on the imaging plane to achieve panoramic three-dimensional stereo measurement [7]. Ortega et al. proposed a combination of ring laser and conical mirror surface. This method can effectively obtain panoramic three-dimensional information, but the combination of laser source and mirror surface is more demanding. And. because its sensor design adopts parabolic catadioptric imaging, parabolic mirror catadioptric imaging has the advantages of simple imaging algorithm and no special geometric corresponding requirements during installation [8].

Through the comprehensive application of Flex and PV3D technologies, the paper constructs a three-dimensional virtual campus system based on panoramic images. The system has good interactivity and users can roam freely in it, so that users have a more realistic and immersive feeling. It has had a profound impact on the school's external publicity and has important promotion and application value.

## 3. Digital 3D Multimedia Panoramic Visual Communication Technology Based on Virtual Reality

Virtual reality is a three-dimensional virtual reality environment created by modern computer technology. In a virtual reality environment, users can participate in the virtual environment through work and better understand what they see and hear. Computer virtual reality technology provides users with an interactive virtual reality environment, in which they can self-manage and actively interact with objects, so as to form a universal experience combining vision, hearing, and touch. In fact, virtual reality requires a deep understanding of cognition, independence, and interaction in applications. The combination of the two enables users to create virtual reality-like concepts, namely, the three key concepts of virtual reality: interaction, understanding, and imagination, as shown in Figure 2. Therefore, it is convenient to improve immersion and improve the ability to interfere autonomously. Instructions for improving virtual reality are given in the study by [9].

### 3.1. Immersion

Immersion is the immersive feeling that the virtual environment in virtual reality technology brings to people. Immersion is also the main criterion for measuring the construction of a virtual reality environment. It is also the main basis for people to obtain a “sense of conception” in experiencing virtual reality technology [10].

### 3.2. Interactivity

Interactivity is the main feature that distinguishes virtual reality technology from traditional 3D animation. When watching 3D animation, the viewer is in a passive state of acceptance [11] and the interactivity of virtual reality allows people to interact with the virtual reality environment and objects. Then, after the color separation filter filters, only the specified wavelength range of light is allowed to pass through. In the virtual reality environment, the viewer is no longer a bystander who passively receives information but can also participate in it.

### 3.3. Autonomy

Autonomy refers to the main characteristics of virtual reality browsing. In the virtual reality environment, users can browse or change the virtual reality environment according to their own intentions.

### 3.4. Panoramic Visual Communication Technology

In summary, the color of the object recognized by the observer is determined by the spectral composition of the light source, the reflection characteristics of the surface of the object, and the observer's sensitivity to the spectrum. Based on the above analysis, this paper further proposes an active vision system model based on the framework of the active vision system [12].

First, each photosensitive unit (that is, pixel) of the CCD will generate a photoelectric effect under the action of the incident light and store a certain amount of photoelectrons corresponding to the light intensity on each photosensitive unit. Generally speaking, this process is characterized by a coefficient, which means that a photon generates several photoelectrons correspondingly. But in fact, the CCD may work in the fat zero mode and each unit has a small number of photoelectrons, which is equivalent to a bias. There are also some noise effects, which are generally not completely linear.

The camera model describes the process of photoelectric conversion. CCD (charge coupled device) is an important device that undertakes the task of photoelectric conversion. It has photosensitivity and the ability to store charges. When the surface feels light, it will generate corresponding charges. First, external light is concentrated through a tiny lens to improve daylighting. The color separation filter then filters the light, allowing only the desired wavelength range of light to pass through; finally, the photosensitive layer converts the light signal through the color separation filter into an electrical signal. The incident light after digital camera CCD can be expressed by the following formulas:

(1) $$\begin{array}{c} R=\int_{0}^{\infty }f_{R}\left(\lambda \right)I\left(\lambda \right)d\lambda , \end{array}$$

(2) $$\begin{array}{c} G=\int_{0}^{\infty }f_{G}\left(\lambda \right)I^{\prime }\left(\lambda \right)d\lambda , \end{array}$$

(3) $$\begin{array}{c} B=\int_{0}^{\infty }f_{B}\left(\lambda \right)I^{\prime }\left(\lambda \right)d\lambda . \end{array}$$

Here, ∫_0_^*∞*^*f*_*R*_, ∫_0_^*∞*^*f*_*B*_, and ∫_0_^*∞*^*f*_*B*_, respectively, represent the wavelength spectrum sensitivity of the camera's three-channel color filter, and the authors represent the intensity of light reaching a certain wavelength of the camera. The wavelength spectrum sensitivity of a digital camera is generally provided by the CCD/CMOS production company. It is the product of the filter function of the color filter and the responsiveness of the photosensitive layer.  Figure 3 shows the response curve of the CCD of a certain digital camera to the spectrum.

Theoretically, it is believed that the response characteristic of CCD to light energy is linear; that is, there is a linear relationship between the amount of exposure and the gray value of the digital image. In fact, neither CCD nor CMOS is completely linear in the process of converting optical signals into electrical signals [12]. The literature pointed out that in an environment where a color camera is used as a precision measuring instrument, it is necessary to solve this problem through photoelectric response linear correction.

The luminous flux received by different areas of CCD/CMOS under a uniform light field is not the same. The luminous flux received at the center of the lens is greater than the luminous flux received around the lens. The literature points out that for different lenses and corresponding focal lengths, it is necessary to use an integrating sphere for shimming correction. In the active vision system model of this article, the above factors have not been considered [13–16].

Assuming that there is only diffuse reflection on the surface of the object, the relationship between reflected light *I*′(*λ*) and incident light *k*(*λ*) can be shown in the following equation:

(4) $$\begin{array}{c} I^{\prime }\left(\lambda \right)=I^{\prime }\left(\lambda \right)\cdot k\left(\lambda \right). \end{array}$$

Here, *I*′(*λ*) represents the intensity of incident light at a wavelength of *λ* at the time *t* and *k*(*λ*) is the reflection coefficient of the material at a wavelength of *λ*. On this basis, to increase the consideration of specular reflection, it is necessary to increase the respective weights of the specular reflection component and the diffuse reflection component. At this time, formula (4) will be rewritten as the following formula:

(5) $$\begin{array}{c} I^{\prime }\left(\lambda \right)=m_{d}I^{\prime }\left(\lambda \right)\cdot k\left(\lambda \right). \end{array}$$

The different TVS and different primary colors used by the projector (such as phosphors) must first know their coefficients in standard chromaticity coordinates to obtain the matrix conversion. Thus, after receiving the signal (if the signal is defined by standard chromaticity coordinates), we must wait until the three primary colors are compared to the corresponding light as the color through transformation.

The projection equipment used in this paper is a panoramic color light source generator (PCSLG) with a transmitting point. The color characteristics of the lighting should be related to the tilt angle, as shown in Figure 4.

In the actual situation, there is a difference between the theoretical projection and the real projection at a certain projection angle due to the manufacturing process. In order to overcome the existence of this difference, the panoramic color structured light generator needs to undergo chromaticity calibration before the actual measurement [17]. The chromaticity calibration will be introduced in the light source color correction algorithm later.

## 4. Realization of the Virtual Campus Roaming System

The virtual campus provides the most intuitive form of campus landscape and facilities, facilitates users' access to campus information, and promotes the construction of universities and the development of distance teaching. The virtual campus is based on high-tech such as geographic information technology, virtual reality technology, and computer network technology, combining campus geographic information with other campus information. Browsing and querying the landscape and information of the ridge garden can be realized through the virtual reality scene interface, and they can be uploaded to the computer network and provided for remote access.

### 4.1. Demand Analysis and Design of the Virtual Campus Roaming

Taking into account the actual roaming needs of users, the basic functions provided by the system include the following parts: viewpoint options, interaction methods, roaming methods, scene selection, and campus introduction as shown in Table 1.

The composition of the roaming panoramic campus is organized by the relative spatial relationship of each panoramic image node in the entire scene. Therefore, in the design and production of the main interface of the panoramic campus roaming, the campus three-dimensional navigation map is used as the basis [18], and then based on it, we place the corresponding object for the reference. And, through the production of command buttons on important campus buildings, the connection of the secondary page is carried out and finally the campus is roamed through the navigation and hotspot connection. The basic framework of campus roaming is shown in Figure 5.

The realization of panoramic roaming interactive technology usually includes three aspects: first, the collection and creation of panoramic images of each element of the site [19]; second, processing of panoramic roaming space; third, design and building of panoramic browsing interface. The acquisition and creation of panoramic images is an important technology in the development of the panoramic roaming school. In the previous section, we discussed and analyzed the key concepts of panoramic design and the application of modern technology. In addition, the transformation of the panoramic roaming site is an important part of the design of the panoramic roaming system. By modifying the panoramic roaming space, 3d panoramic images of various locations can be integrated into the virtual roaming space for viewers to walk freely. The design and manufacture of the panorama browsing interface [20] are used by the audience when viewing the panorama website. Therefore, the design and construction quality of the browsing interface affect the completion of three-side panoramic roaming interaction. The best panorama browsers are designed to make it easy for viewers to view their favorite virtual scenes.

### 4.2. Experimental Steps

1. Use an ordinary digital camera to acquire material images; a total of 20 groups are acquired, and the number of material images in each group increases sequentially, which are 5, 6, ..., 26.
2. Carry out cylindrical projection on the acquired material images, and calculate the camera horizontal angle of view (hfov) and camera pixel focal length (f) of 20 groups of material images.
3. For two adjacent images in the same scene, use the SIFT-based image matching algorithm and the Harris-based image matching algorithm to detect and match feature points and record the number of detected feature points and the matched feature point pair quantity [21].
4. Perform coordinate transformation on the image to be spliced through the matching feature point pairs to complete the image splicing. Through the above steps, the data obtained is shown in Table 2. Among them, detection represents the number of detected feature points, match represents the number of matched feature point pairs, hfov represents the camera's horizontal viewing angle, and f represents the camera pixel focal length [22].

### 4.3. Experiment Analysis

Through the analysis of the above experimental data, we can know that multiple feature point pairs can be matched together in multiple data images in the same scene. In the same case, the SIFT algorithm has more special integration points than the Harris algorithm, as shown in Figure 6. The special points obtained by the SIFT feature extraction algorithm include dozens of error points from Harris corner. The extraction algorithm [23] also includes noncolor elements in the graph.

Estimation of surface spectral reflectance of objects: because it is very difficult to directly calculate the surface spectral reflectance of objects, in consideration of the time of the active vision system, this paper uses three-channel reflectance instead. Solutions: experiments show that using three-channel interference to adjust the color of the product can reduce the accuracy by 44% to 11% and achieve better results. However, when calculating the effects of the three methods in light or standard white light, there may be slight differences due to differences in the intensity of the projected light. Therefore, how to develop an environmental model to solve the three-channel concept is a necessary condition for further research [24].

In addition, the material surface with special strong specular reflection will cause the light saturation phenomenon of the digital camera, which will affect the separation of specular reflection components and the location of diffuse reflection objects. Therefore, in a wide range of applications, attention should be paid to adjust the aperture size and exposure time of digital cameras or adopt wide dynamic camera technology.

## 5. Conclusion

The application system of this article simply takes a school as an example, and the amount of data is relatively small. However, in some commercial applications, the amount of image data in a three-dimensional virtual environment is often very large. Image storage and indexing technology is a key point of virtual roaming. Combining database technology for image storage and retrieval is a direction worthy of further research. Interactive roaming is a complete roaming process. An exploration of the interaction and interactive nature of 3d virtual travel systems is also worth listening to. How to create an interactive way that is related to the audience's works and does not affect the audience's sense of reality is a suitable research direction. In the display of high-resolution images, how to use a variety of display technologies to produce beautiful and fast images is also an undetermined problem of the system, which should be further studied in the future. In short, the research of 3D virtual roaming technology has important theoretical significance and application value. The research and discussion on it in this paper are far from enough. In the follow-up research, on the basis of the existing research, we should continuously absorb various new related technologies and methods, further deepen the research, and achieve better results for the panoramic display and apply it to a broader field.

In a word, the research of 3D virtual tourism technology has important theoretical value and application value. The research and discussion in this paper are far from enough. In future research, on the basis of existing research, many new technologies related to the process should be further extended to in-depth research, to achieve the best effect of panoramic images and apply them to wider fields.

## Figures and Tables

**Figure 1:** Three-dimensional animation interaction.

**Figure 2:** The main characteristics of virtual reality.

**Figure 3:** The response curve of the camera spectrum.

**Figure 4:** Correspondence between PCSLG's hue value and projection angle.

**Figure 5:** Schematic diagram of the interactive roaming framework structure.

**Figure 6:** Feature point pairs matched by the SIFT algorithm and Harris algorithm.

**Table 1:** Function summary table of virtual campus roaming system.

Viewpoint control	Best: move the viewpoint to the most suitable observation position when switching the panorama.
Interactive operation	Mouse: use the mouse of the computer as the main input device to complete the panoramic image viewing and interactive roaming functions.
Scene switching	Map navigation: switch to the corresponding panoramic scene view through the hotspot setting connection of the place.
Campus profile	Campus introduction: a brief introduction to the whole campus, so that the viewer has an overall understanding of the school.

**Table 2:** Experimental result data.

	5				6			
	Detection	Match	hfov	f	Detection	Match	hfov	f

SIFT	1575/1506	7	1.23	442.13	1647/1653	6	1.23	553.6
Harris	902/632	6	2.31	440.23	988/632	6	1.56	253.12
	7				8			
	Detection	Match	Hfov	f	Detection	Match	Hfov	f

SIFT	1802/1653	9	0.93	665.23	1758/1236	49	0.86	775.36
Harris	956/231	5	0.8	563.59	953/856	6	0.89	652.39

## Data Availability

The data used to support the findings of this study are available from the corresponding author upon request.
